# Analysis and Prediction of Influence Factors of Green Computing on Carbon Cycle Process in Smart City

**DOI:** 10.1155/2022/7546742

**Published:** 2022-08-08

**Authors:** Xianghua Huang, Shidong Chen, Decheng Xiong, Chao Xu, Zhijie Yang

**Affiliations:** ^1^School of Geographical Sciences, Fujian Normal University, Fuzhou 350007, China; ^2^Sanming Experimental Forest, Sanming 365001, China

## Abstract

Global warming has become the focus of attention of the international community, and the control of carbon dioxide emissions has become one of the necessary choices for the development strategies of countries around the world. Cities are places where carbon dioxide emissions are concentrated. The key to controlling carbon emissions is to control the carbon emissions of cities. My country is currently in the process of rapid urbanization. Quantitative studies of the carbon cycle at the city level will help to take stock of carbon dioxide emissions in cities. On the other hand, it is helpful to understand the status and role of the urban carbon cycle in the process of the regional carbon cycle. Through the analysis and prediction of the elements influencing the carbon cycle of smart cities, this paper first determines the factors affecting smart cities in the carbon cycle process as industrial carbon emission strength factors, industrial structure effects, economic development factors, and population elements. It is found that the major positive factors affecting the significant add of CO2 emissions in smart cities from 2010 to 2019 are economic development factors and demographic factors, including economic development factors GDP/per capita GDP. The per capita contribution to CO2 emissions is higher than the model established by adjusting the affecting elements of overall CO2 emissions, except that the proportion of economic development factors in total CO2 emissions from 2013 to 2015 was lower than the increase in total CO2 emissions. The comparison can better reflect the relation between CO2 emissions and influencing elements. The main determinants affecting CO2 emissions are the expansion of the financial condition, the increase in the average daily population, and the increase in construction work. The adaptation index is judged to be consistent, indicating that the model adjustment effect is good; finally, the green computing in the smart city predicts the carbon cycle process, and the actual value trend line and the predicted value trend line are not much different from the practical value, the forecast error is small, and the prediction results are credible. Global warming has become the focus of attention of the international community, and carbon emission control has become one of the necessary options in the development strategies of countries around the world. Cities are the places where carbon emissions are concentrated. The key to controlling carbon emissions is to control urban carbon emissions. At present, my country is in the process of rapid urbanization. Quantitative research on the carbon cycle at the city level will help to establish an inventory accounting of urban carbon emissions. On the other hand, it is convenient to deeply understand the status and role of the urban carbon cycle in the process of the regional carbon cycle.

## 1. Introduction

The cost of electricity varies from plant to plant, and each plant emits a different amount of carbon for every certain amount of electricity produced. Traffic for this infrastructure service can come from anywhere in the world. Due to latency, it is desirable to path traffic to the data center that is geographically proximate, has the lowest cost of electricity, and emits the least amount of carbon dioxide per request. Achieving all of these goals is not always possible, so the network and compute modules of the base station have been modeled as a figure and a proposed stratus system that uses Voronoi partitioning to decide which data center should be given to the cloud due to relatively priority communicate to the operator [1]. The purpose of load balancing is to reduce resource consumption and reduce the consumption efficiency required by cloud computing. This confirms the need for new measures to balance energy efficiency, energy consumption, and carbon emissions in the cloud. The article discusses cloud load balancing techniques and further compares them based on various parameters using the different techniques considered such as performance, scalability, and associated overhead. [2]. Green computing refers to the practice of using computing resources more efficiently while maintaining or improving overall performance. Sustainable IT services require the integration of green IT practices such as energy management, virtualization, improved cooling technologies, recycling, e-waste disposal, and IT infrastructure optimization to meet growth demands. Recent research shows that IT departments can cover nearly 50% of a company's total energy costs for electricity, review the supporting IT literature, build interest, and identify a set of core principles for designing sustainable IT services [3]. The advent of Mobile Cloud Computing (MCC) technology, which enables mobile users to use cloud computing in an environmentally friendly manner, is an effective strategy to meet the needs of today's industry. But, the limitations of wireless network bandwidth and equipment bandwidth pose some obstacles to the implementation of MCC which are additional power consumption and delay. To solve this problem, there is a dynamic mobile cloud computing (DECM) model, which focuses on handling the extra power consumption during wireless communication by using a dynamic cloud-based model (DCL) and validates models by simulating real-world scenarios and providing reliable evaluation results. The first study addresses the problem of energy waste in a dynamic network environment; second, the proposed model provides direction and theoretical support for future research [4]. One of the challenges of cloud computing is frequent optimization of cloud servers, mainly focusing on load balancing in cloud data centers to improve host performance and reduce the number of active hosts to support the concept of green computing for a fee. To balance the weight of the data center, migration equipment is required so that virtual machines can be migrated from an overloaded army to a lighter army. This document provides Threshold-Based Dynamic Balancing Optimization and Algorithm (DCABA) for cloud servers. Unlike traditional server optimization strategies that only trade off the scale and balance of map resources used by CPU, RAM, and BW on physical servers, DCABA also reduces the number of active hosts that can reduce cloud service costs. The cost of services in the cloud industry can be reduced through efficient use of available resources [5] and research of the law of calculating carbon emissions based on the physicochemical stage. According to the characteristics of green buildings, life cycle analysis (LCA) is used to quantitatively analyze the CO2 emissions of buildings. Vensim (system dynamics software package) is used to analyze the carbon emissions in the physicochemical phase, identify the main subsystems that affect carbon emissions, and extensively consider the differences in carbon dioxide emissions of each subsystem under different construction technologies. In the physical and chemical emissions trading mechanism, the total amount of emissions trading remains unchanged, and the market price of each subsystem is adjusted. In this case, it is recommended to gradually increase the price calculation coefficient. By introducing a pricing system, construction companies are encouraged to use high-efficiency emission reduction technologies; at the same time, the system is also used to establish an emission rights trading system, which accelerates the process of energy conservation and emission reduction in China and the world [6]. An Integrated Sustainable Waste Management System (IWMS) is now a priority as it contributes to the EU 2020 strategic goals. New web-based technologies can now be used to monitor, manage, and analyze spatially distributed systems through processes. There is an increasing focus on applying these technologies to the production of systems and utilities to provide flexibility and efficiency. The main objective of the DSS is to reduce the net CO2 emissions from the IWMS, and a comparative analysis of the improvement of independent acquisitions of the entire IWMS was carried out using the model in a medium-sized city in southern Italy. The results in each case show a multiflow aggregation system for the dry discontinuous and a single-flow circulation system for the organic and glass sections. At the same time, various combinations of methods and information were found in both cases [7]. The carbon footprint of the global communications network was estimated at 2% in 2007 and is expected to increase to 4% by 2020. By choosing efficient and environmentally friendly hardware and software, you can reduce your carbon footprint, save money, and increase the reuse of utility poles. A lot of research has been done around the world to promote and optimize people's productivity at the industry level. With the goal of creating a sustainable industry for future generations, reducing carbon dioxide emissions, and developing sustainable energy, it is necessary to measure, model, and predict the energy consumption of institutions with different computing resources and resources [8]. The planet is very sensitive to climate change, and the impact of climate-related natural disasters will increase. By 2050, nearly 70% of the world's population will live in cities, and climate flexibility policies will become increasingly important. According to selected case studies, energy efficiency, low-carbon green urban design, and assessment of the impact of urbanization on the environment and climate change are considered complementary tools for addressing climate resilience. By combining climate-friendly economic policies, sustainable cities, and traditional low-carbon green approaches with climate-flexible and smart city development, cheap carbon can deliver greater benefits at lower prices [9]. This paper analyzes the CO2 emissions of China's secondary industry from 2000 to 2015 and uses CO2 emissions as the environmental impact assessment standard. Research on the secondary industry shows that carbon emissions account for a large proportion of total carbon emissions, but the growth rate has slowed down. From the stock model, the elastic carbon emission factor is estimated by time series analysis, indicating that technology has a significant impact on reducing energy intensity, that is, reducing energy consumption per unit of added value will have a positive impact on reducing carbon emissions. The GM secondary industry emission model (1.1) is used for analysis and prediction from 2016 to 2020, to analyze the growth links of CO2 emissions, and to provide a scientific basis for economic decision-making [10]. Based on system dynamics, environmental approaches, CO2 trends, CO2 concentrations, and temperature changes over the next 50 years are simulated using a macroscopic approach. Empirical analysis finds that anthropogenic carbon dioxide emissions are the main factor influencing these trends. The results suggest that the proposed Paris Agreement could achieve −3.2% CO2 reduction. From there, future global carbon reductions and their investments are calculated and described, and reports are provided to relevant authorities on carbon reduction plans [11]. The response grey analysis analyzes the relationship between Beijing's economic growth, energy consumption structure, industrial structure, population size, urbanization and pollution intensity, and carbon dioxide emissions from 2003 to 2012. If the relevant factors remain at the current level, carbon dioxide emissions will continue to increase in the future. Finally, significant changes in industrialization structure, industrial density, urbanization, economic development, population size and corresponding factors, emission reduction measures, and recommendations are presented [12]. Through correlation and regression analysis, a comprehensive relationship between carbonate emissions and runoff factors was established, and the main factors were successfully developed from 16 preferred factors such as GDP, total population, total energy consumption, and industrial production. Then, the least-squares parameters of the support vector machine are optimized using the subgroup algorithm. By using an optimized predictive model, passenger aircraft parameter selection overcomes the difficulties of least squares support, increasing the overall speed of learning and investigation. The results show that the accuracy of CO2 emission prediction is indeed improved [13]. This paper takes Qingdao as a research institution to discuss carbon footprint and its factors affecting production, transportation, construction, and total emissions. Based on the analysis of the relationship between Qingdao's populations, economy, industrial demand, and carbon dioxide emissions, the globalization theory is used to predict the trend of carbon dioxide emissions under three different scenarios [14]. Based on previous research, 12 factors affecting China's construction industry have been identified as being related to carbon emissions. Taking the indicator data from 2000 to 2016 as an example, the strong correlation effects of 8 factors are filtered according to the initial grey relational analysis. The CO2 model combined with the BP neural network provides a network prediction model for the Chinese construction industry. Neural networks are used to predict CO2 drivers, forecasting projected CO2 emissions from 2017 to 2020. Research shows that sample predictions are consistent with the situation itself, indicating that training the network generically is effective. Some influencing factors appear to have a large impact on building CO2 emissions and can be used to predict building CO2 emissions. This predictive model improves the training speed of neural networks and provides a new tool for predicting CO2 emissions [15].

## 2. The Carbon Cycle Process of Smart Cities

### 2.1. Smart City Ecosystem

The urban ecosystem is mainly composed of green plants and humans as producers, other animal species and humans as consumers, various microorganisms and small animals as decaying matter, and the government and residents as security coordinators. As shown in Figure 1, in the composition of the urban ecosystem, governments at all levels and residents play an important role in providing the structure, function, and service functions of the urban ecosystem and are an important factor in ensuring the harmonious development of the city. Of course, urban ecosystems are different from natural ecosystems and have obvious characteristics: First, urban ecosystems are ecosystems with man-made environments as their main components. It is people with human intelligence who create cities through work, and the development of urban ecosystems is inseparable from human control and behavior. In contrast to natural ecosystems, the main organs of their living systems are humans, not other animals, plants, and microorganisms. Frequent human activities promote the well-being of urban ecosystems but also alter the natural environment by consuming large amounts of energy and materials, making cities the most polluted places. Second, the urban ecology is not perfect. The natural ecosystems of cities are gradually being replaced by artificial ecosystems. Animals, plants, and microorganisms in natural ecosystems have lost their natural habitats to survive in cities, urban biomes are shrinking, and urban ecosystems are severely flawed. The number of green plants in the “producers” of urban ecosystems is decreasing, and their role in cities has become to beautify the urban landscape, purify the air, and reduce pollution. Third, the urban ecosystem is an open, diverse, and dependent ecosystem. The urban ecosystem cannot provide all the energy and materials it needs, and the materials and energy produced by producers are far from meeting the needs of consumers and are completely dependent on the input of external systems.

### 2.2. Carbon Cycle Characteristics of Smart City Eco-economic System

The carbon cycle process in the urban eco-economic system is obviously different from that in the natural ecosystem. Therefore, it is necessary to understand the characteristics of the carbon cycle process in the green urban economic system as a whole. As a complex and interdependent socio-economic system, the carbon cycle in a green urban economy is characterized by high complexity, uncertainty, and spatiality. The main manifestations of heterogeneity are as follows: first, there is a large-scale carbon exchange between the urban green economic system and the outside world. Carbon cycle processes cover parts of the urban footprint and even affect biogeochemical processes in larger areas. The spatial extent of the impact depends primarily on the city's coal flow and transportation modes. Secondly, the urban carbon cycle includes natural processes and man-made processes, mainly man-made processes; the carbon cycle of the artificial part of the city is mainly affected by human factors while the carbon cycle of the natural part is mainly driven by natural processes. The carbon cycle consists of horizontal and vertical carbon flows. Among them, the horizontal carbon flow is dominated by human-made processes, and the vertical carbon flow includes both human-made and natural processes. Fourth, the carbon cycle of the urban eco-economic system exhibits great spatial heterogeneity. The intensity, quantity, and speed of urban carbon flow depend on the type and level of urban social development, urban function, industrial type, economic structure, energy structure, and social factors such as energy efficiency, human activities, and anthropogenic carbon storage such as carbon storage in vegetation and soil and carbon dioxide storage in public buildings and dwellings (wood, furniture and carbon storage, books) as shown in Figure 2.

1. The urban ecological economic system has a huge carbon exchange with the outside world, and the spatial scope of its impact mainly depends on the urban carbon metabolism flux and the mode of transportation.
2. The urban carbon cycle process includes natural processes and man-made processes, with man-made processes as the main process; the carbon cycle process in the artificial part of the city is mainly affected by human factors while the carbon cycle process in the natural part is mainly controlled by natural processes.
3. The carbon cycle of the urban ecological economic system includes two parts: horizontal and vertical carbon flux.
4. The carbon cycle of the urban ecological and economic system has great spatial heterogeneity. The intensity, scope, and rate of urban carbon flux depend on the mode and level of urban social development, urban functions, industrial types, economic structure, and energy structure and energy social factors such as usage efficiency.
5. Affected by human activities, the urban ecological economic system also has a certain anthropogenic carbon pool, such as the carbon storage of urban green vegetation and soil and the carbon storage of urban buildings and households.

### 2.3. The Impact of Smart Cities on the Carbon Cycle Process

As a region where human economic activities are concentrated and fossil fuels are burned, the human economic activities and energy consumption of cities lead to a large amount of carbon dioxide emissions. Meanwhile, compared with natural ecosystems, the carbon cycle of the urban green economy is a complex system involving natural and anthropogenic processes, horizontal and vertical processes, and economic and chemical processes. Due to gender and spatial heterogeneity, urban carbon cycle processes are more complex and diverse. So far, research on the carbon cycle has mainly focused on natural ecosystems such as forests, grasslands, and soils. From the perspective of human activities affecting global climate change, urban systems are undoubtedly one of the most important links in the global carbon cycle. The effectiveness of the circulation mechanism is directly related to the depth and magnitude of human impacts on climate change. China is in a stage of rapid economic development. With the acceleration of urbanization in my country and the proliferation and expansion of cities, the impact of the urban carbon cycle (especially anthropogenic carbon dioxide emissions) on global and regional climate change is discussed. Studying the carbon cycle process in China's urban system can not only provide a decision-making basis for formulating a national low-carbon city strategy but also provide new methods and approaches for reflecting and reimagining China's urban development model. This is a period of rapid industrialization and urbanization, the economy is growing, but environmental concerns are of paramount importance. In addition, heavy chemical cities, mainly metallurgy and petrochemical, have a large demand for raw materials and energy and are expected to emit high carbon dioxide emissions. Therefore, in the process of economic development, it is also faced with huge resource and environmental constraints.

As a region where human economic activities are concentrated and fossil fuel burning is concentrated, urban human economic activities and energy consumption have brought a large amount of carbon emissions. It is in the period of rapid industrialization and urbanization. The economy is developed, but the environmental problems are prominent. Moreover, cities with heavy chemical industries, mainly metallurgical and petrochemical industries, have a large demand for resources and energy and thus have a large carbon emission expectation. Therefore, in the process of economic development, it is also faced with huge resource and environmental constraints.

### 2.4. Low-Carbon Development of Smart Cities

In recent years, the global greenhouse effect caused by anthropogenic carbon emissions has become a hot topic in the international academic community and governments. China is one of the world's largest carbon dioxide emitters and faces enormous pressure to reduce carbon emissions in international climate negotiations. Therefore, reducing carbon dioxide emissions and sustainable economic and social development have become important topics in my country's economic development, and developing a low-carbon economy has become an inevitable choice for the current economic and social transformation. The first is to explain the connotation of a low-carbon city, explain the concept of a low-carbon city, and scientifically define the boundaries between urban development and land and energy efficiency. The second is to formulate a low-carbon city index quantification system and evaluation standard based on the regional environmental constraint index system and combine it with the urban planning evaluation system. Third, scientific urban planning is the first step in building a low-carbon city. Due to the rigidity of urban planning in my country, it is difficult to change urban planning once it is formulated and implemented. Therefore, low-carbon urban planning and design must ensure dynamic urban development, clean environmental quality, and environmental comfort. Transportation systems, green buildings, and clean and efficient low-carbon energy can lead to a healthy and reasonable lifestyle. Fourth, the industrial development of low-carbon cities requires a low-carbon cycle. Cities are centers of economic growth, and new industrial areas can stimulate economic development and create jobs in cities. Establishing a circular economy and clean manufacturing are the principles and guidelines that should be followed in building a low-carbon city. Fifth, build an environment-friendly transportation system, advocate, and implement public transportation and transportation-oriented transportation methods. Transportation strategies for low-emission cities can be implemented in two ways: controlling the number of clean transportation trips, reducing carbon dioxide emissions, and personal transportation. Sixth, upgrade green buildings. Green building refers to maximizing resource conservation (energy saving, soil protection, water source protection, and material protection) throughout the entire life cycle of a building, protecting the environment, reducing pollution, and providing healthy, useful, and efficient spaces that live in harmony with nature.

1. It is necessary to clarify the connotation of low-carbon city, define the concept of low-carbon city, scientifically define the boundary of urban development, and use land and energy efficiently.
2. On the basis of the regional environment and resource constraints leading index system, establish a quantitative low-carbon city index system and evaluation standard and incorporate it into the urban planning system and evaluation system.
3. Scientific urban planning is the first step in building a low-carbon city.
4. The industrial layout of low-carbon cities should be low-carbon and circular.
5. Constructing a green transportation system, advocating, and implementing public transportation priority and leading transportation modes.

## 3. Green Computing Models

### 3.1. Problem Analysis

The layout and current state of the virtual machine need to be considered when scheduling jobs for the correct type of virtual machine. In the resource allocation model, the predicted and control values of various tasks are first obtained through appropriate prediction algorithms and control strategies, and a reasonable initial allocation of resources is made in combination with the current distribution and status of various types of tasks. To simplify problem analysis, the following reserved definitions are created: for all sets of physical hosts: <host_*j*_ > =(host_1_, host_2_, ⋯, host_*j*_, host_*N*_) and sets of virtual machines: <*VM*_*i*_ > =(*VM*_1_, *VM*_2_, ⋯, *VM*_*i*_, ⋯, *VM*_*M*_), define an *M* × *N* state statistics matrix *A*_*M*×*N*_. Element *A*_*M*×*N*_ in matrix *a*_*ij*_ is defined as the total number of virtual machines of type host_*j*_ running on *VM*_*i*_. The statistics matrix of the virtual machine is as follows.

Scheduling tasks to the corresponding type of virtual machine needs to take into account the distribution and current state of the virtual machine. In the resource allocation model, the predicted and control values of various tasks are first obtained through appropriate prediction algorithms and control strategies, and a reasonable preconfiguration of resources is made in combination with the current distribution and status of the corresponding types of virtual machines.

(1) $$\begin{array}{c} A_{M\times N}=\left(\begin{array}{ccc} a_{11} & \cdots & a_{1N}\\ \vdots & a_{ij} & \vdots \\ M_{1} & \cdots & a_{MN} \end{array}\right),in:i\in \left\{1,\cdots ,M\right\},j\in \left\{1,\cdots ,N\right\}. \end{array}$$

For the set of all physical hosts: 〈host_*j*_〉 and the set of task types: 〈task_*j*_〉, define the average speed matrix *U*_*M*×*N*_. Element *u*_*ij*_ in the matrix is defined as the average speed at which tasks of class task_*i*_ are executed on host_*j*_ (average execution time is 1/*u*_*ij*_). The average rate matrix is as follows:

(2) $$\begin{array}{c} U_{M\times N}=\left(\begin{array}{ccc} u_{11} & \cdots & u_{1N}\\ \vdots & u_{ij} & \vdots \\ u_{M1} & \cdots & u_{MN} \end{array}\right),in:i\in \left\{1,\ldots ,M\right\},J\in \left\{1,\ldots ,N\right\}. \end{array}$$

The overall quantity of physical main engine in the bunch is N. For *n* (*n* ≤ *N*) running physical main engine, the overall quantity of replicas of different types of fictitious machines running on each physical main engine (host_*j*_) is *q*_*j*_, responsible for running their respective task types and virtual machines in active/sleep state. Define the size of state *R*_*ik*_ to indicate whether a virtual machine (type *VM*_*i*_) on the physical host is performing the correct type of task, that is, as follows:

(3) $$\begin{array}{c} R_{ik}=\left\{\begin{array}{cc} 1, & \text{Is running}\\ 0, & \text{In idle state} \end{array}\right.in:i\in \left\{1,\ldots ,M\right\},k\in \left\{1,\ldots ,q_{i}\right\}. \end{array}$$

By analyzing the bunch status and allocation and their corresponding VM types, combined with appropriate prediction algorithms, appropriate premonitoring behaviors can be performed, which can improve the utilization of cloud computing platform resources, lower power depletion, and improve actual performance simultaneously. Improve system response and stability. The control behavior is now defined as follows.

For the set of all physical hosts: 〈host_*j*_〉 and the set of virtual machines: *VM*_*i*_, define a power *M*×*N* on the control matrix Start_*M*×*N*_. Element Start_*ij*_ in the matrix is defined as: host_*j*_ to Start_*ij*_ starting from virtual machines of type *VM*_*i*_. The open control matrix Start_*ij*_ becomes the following representation:

(4) $$\begin{array}{c} {\text{Start}}_{M\times N}=\left(\begin{array}{ccc} {\text{Start}}_{11} & \cdots & {\text{Start}}_{1N}\\ \vdots & {\text{Start}}_{ij} & \vdots \\ {\text{Start}}_{M1} & \cdots & {\text{Start}}_{MN} \end{array}\right),\\ {\text{Start}}_{ij}=\left\{\begin{array}{c} \text{non}-\text{0},{\text{Start Start}}_{ij}\text{ virtual machines of type }VM_{i}{\text{ on host}}_{j}\\ 0,{\text{There is no need to start Start}}_{ij}\text{ virtual machines of type }VM_{i}{\text{ on host}}_{j}\;. \end{array}\right. \end{array}$$

For all physical main engine sets: 〈host_*j*_〉 and fictitious machine type sets: *VM*_*i*_, define a *M* × *N* shutdown control matrix Shut_*M*×*N*_. An element Shut_*ij*_ in the array is defined as shutdown the virtual machine type on host_*j*_. The closing stroke control matrix is expressed as follows:

(5) $$\begin{array}{c} {\text{Shut}}_{M\times N}=\left(\begin{array}{ccc} {\text{Shut}}_{11} & \cdots & {\text{Shut}}_{1N}\\ \vdots & {\text{Shut}}_{ij} & \vdots \\ {\text{Shut}}_{M1} & \cdots & {\text{Shut}}_{MN} \end{array}\right),\\ {\text{Start}}_{ij}=\left\{\begin{array}{c} \text{non}-\text{0},{\text{Close Start}}_{ij}\text{ virtual machines of type }VM_{i}{\text{ on host}}_{j}\\ 0,{\text{There is no need to close Start}}_{ij}\text{ virtual machines of type }VM_{i}{\text{ on host}}_{j}\;. \end{array}\right. \end{array}$$

In the cloud computing system model proposed in this chapter, for all sets of physical hosts: 〈host_*j*_〉 and *VM*_*i*_, the overall quantity of fictitious machines that need to be controlled to be shifted on or off during a certain resource provisioning process is delimited as *y*_i,start_′, *y*_*i*,shut_′ respectively.

(6) $$\begin{array}{c} \left\{\begin{array}{c} y_{i,\text{start}}^{\prime }=\sum_{j=1}^{N}{\text{Start}}_{ij}\\ y_{i,\text{shut}}^{\prime }=\sum_{j=1}^{N}{\text{Shut}}_{ij} \end{array}.\right.. \end{array}$$

### 3.2. Many Goals Constrained Majorization Model

From the above discussion, it can be concluded that the power consumption of a cloud computing platform mainly depends on the quantity of powered main engine and fictitious machines, and frequent power on and off will also cause huge additional strength consumption. Thus, the energy depletion of the cloud computing platform can be expressed as

(7) $$\begin{array}{c} E=E\left(n,a_{ij}\right)+E\left(\Delta V,\Delta H\right). \end{array}$$

Below *E*(*n*, *a*_*ij*_) shows the stable power consumption generated by the host and the driven virtual machine, *E*(Δ*V*, Δ*H*) shows the additional control power consumption caused by switching between the virtual machine and the physical host, Δ*V* shows the control worth of the virtual machine, and Δ*H* shows the control worth of the host. Allocating the necessary resources to as few hosts as possible improves energy efficiency and reduces power consumption. In this chapter, you can disable and, if necessary, enable redundancy when modifying virtual machines to improve the overall energy efficiency of the bunch.

The useable resources of each physical main engine are abstracted as a two-dimensional vector: host_*j*_ : (MIPS_*j*_^remain^, Mem_*j*_^remain^); MIPS_*j*_^remain^, and Mem_*j*_^remain^ are host_*j*_'s available CPU resources and available disk space, respectively. A vector space analysis looks like this:

MIPS_*j*_^remain^ represents the available CPU resources to host_*j*_, and Mem_*j*_^remain^ shows the memory airspace useable to host_*j*_.

The host storage space (memory, mem) determines the number of virtual machines that the host can run simultaneously, i.e., if there is not enough memory, no more virtual machines can be started. The sum of the memory allocated to all virtual machines cannot exceed the physical host's memory limit. Host CPU cores are shared by all virtual machines. This chapter modifies the time-sharing policy kernel of virtual machines to assign time slots to each virtual machine. All virtual machines run at a CPU peak that does not exceed the capacity of the host. This chapter uses MIPS (Million Instructions Per Second) to measure CPU performance; the sum of MIPS allocated to all virtual machines cannot exceed the MIPS limit of the physical host CPU. Therefore, a two-dimensional vector is chosen: host_*j*_ : (MIPS_*j*_^remain^, Mem_*j*_^remain^) as the source space of the physical host. Each virtual machine also selects a two-dimensional vector: *VM*_*i*_ : (mips_*i*_, men_*i*_) if the demand for virtual machine resources, i.e., host_*j*_ : (MIPS_*j*_^remain^, Mem_*j*_^remain^), *VM*_*i*_ : (mips_*i*_, men_*i*_). In summary, the studied problem has been established as a multicriteria optimization model with constraints, and its mathematical form is as follows:

(8) $$\begin{array}{c} E\left(n,a_{ij}\right)=\sum_{j=1}^{N}\left[p_{j}^{host}+q_{j}\times p_{j}^{vm}\right]\times t,q_{j}=\sum_{i=1}^{M}a_{ij}. \end{array}$$

In Equation (8), *E*(*n*, *a*_*ij*_) shows the stable strength consumption generated by activated main engine and fictitious machines, which is proportional to the total quantity of activated main engine in cluster *n* and the sum of different types of fictitious machines activated on each host.

*E*(*n*, *a*_*ij*_) represents the stable energy consumption generated by the main engine and fictitious machines that are turned on, which is proportional to the total quantity of main engine *n* that are revolved on in the cluster and the total quantity of fictitious machines that are turned on in each host *q*_*j*_, *p*_*j*_^host^ and *p*_*j*_^*vm*^ represent the strength consumption of the main engine host_*j*_, and each virtual machine turned on requires increased power consumption.

(9) $$\begin{array}{c} E\left(\Delta V,\Delta H\right)=\sum_{j=1}^{N}\sum_{i=1}^{M}{\text{Start}}_{ij}\times \Delta p_{j}^{vm\text{Start}}\times \Delta t_{j}^{vs\text{Start}}\\ +\sum_{j=1}^{M}\sum_{i=1}^{M}{\text{Shut}}_{ij}\times \Delta p_{j}^{vm\text{Start}}\times \Delta t_{j}^{vs\text{Start}}\\ +\sum_{j}\Delta p_{j}^{\text{hostStart}}\times \Delta t_{j}^{\text{hostStart}}\\ +\sum_{j}\Delta p_{j}^{\text{hostShut}}\times \Delta t_{j}^{\text{hostShut}}. \end{array}$$

In Equation (9), *E*(Δ*V*, Δ*H*) represents the extra control power consumption caused by switching between the virtual machine and the physical host, ∑_*j*=1_^*N*^∑_*i*=1_^*M*^Start_*ij*_ × Δ*p*_*j*_^vmStart^ × Δ*t*_*j*_^vsStart^ is equal to the extra control power consumption caused by the virtual machine opening process, ∑_*j*=1_^*N*^∑_*i*=1_^*M*^Shut_*ij*_ × Δ*p*_*j*_^vmStart^ × Δ*t*_*j*_^vsStart^ is equal to the extra control power consumption caused by the switching, and the virtual machine shutdown process is generated; ∑_*j*_Δ*p*_*j*_^hostStart^ × Δ*t*_*j*_^hostStart^ is equal to the host that started the process. The additional control power ∑_*j*_Δ*p*_*j*_^hostShut^ × Δ*t*_*j*_^hostShut^ produced is equal to the additional control power produced by shutting down the host process. Δ*p*_*j*_^vmStart^, Δ*t*_*j*_^vsStart^, Δ*p*_*j*_^vmStart^ and Δ*t*_*j*_^vsStart^ represent the instant startup performance of the virtual machine, the startup time of the virtual machine, the instant shutdown performance of the virtual machine, and the shutdown time of the virtual machine on the host machine, Δ*p*_*j*_^hostStart^, Δ*t*_*j*_^hostStart^ and Δ*p*_*j*_^*hostShut*^, respectively, represent the instant startup of the performance host, when the host was turned on or off.

Δ*p*_*j*_^vmStart^, Δ*t*_*j*_^vsStart^, Δ*p*_*j*_^vmStart^, and Δ*t*_*j*_^vsStart^, respectively, represent the instantaneous power of opening the virtual machine, the time of opening the virtual machine, the instantaneous power of closing the virtual machine, and the time of closing the virtual machine on the host host_*j*_; Δ*p*_*j*_^hostStart^, Δ*t*_*j*_^hostStart^, Δ*p*_*j*_^hostShut^, and Δ*t*_*j*_^hostShut^ represent the instantaneous power of opening the host host_*j*_, the opening time, the instantaneous power of closing the main engine, and the time of closing the main engine, separately.

(10) $$\begin{array}{c} \sum_{i=1}^{N}{\text{Start}}_{ij}=y_{i,start}^{\prime }. \end{array}$$

Constraint (10) states that the overall quantity of open fictitious machines of the corresponding type is fair to the quantity of open fictitious machines.

(11) $$\begin{array}{c} \sum_{i=1}^{N}{\text{Shut}}_{ij}=y_{i,\text{shut}}^{\prime }. \end{array}$$

Constraint (11) means that the total number of virtual machines of the corresponding type to be shut down is equal to the number of virtual machines to be shut down;

(12) $$\begin{array}{c} \sum_{i=1}^{N}\left[{\text{Start}}_{ij}\times {\text{mem}}_{i}\right]\leq {\text{Mem}}_{j}^{\text{remain}}, \end{array}$$

(13) $$\begin{array}{c} \sum_{i=1}^{N}\left[{\text{Start}}_{ij}\times {\text{mips}}_{i}\right]\leq {\text{MIPS}}_{j}^{\text{remain}}. \end{array}$$

Constraints (12) and (13), respectively, specify the constraints on virtual machines by the available CPU and Mem resources of physical hosts in the cluster.

### 3.3. Prognostication and Control

So as to enable resource allocation to continuously satisfy the resource demands of various tasks and avoid the problem that resource allocation lags behind user requests, it is necessary to predict the arrivals of various tasks in the next cycle. For different task types, forecast periods, and application scenarios, different forecasting algorithms need to be selected, such as exponential smoothing, period analysis, trend extrapolation, and Markov forecasting models. This chapter adopts the cubic exponential smoothing algorithm to predict the size of the corresponding type of load. The small prediction period should depend on the implementation time of the task, the algorithm time-consuming, the power-on/off time of the physical host and the virtual machine, and other factors. If the selected prognostication period is too brief, it will have a great impact on the stability of the system, and at the same time, it will increase the cost of system control energy consumption. Cloud computing service providers can reasonably choose the size of the forecast period in the light of different situations.

Assuming that the system is currently in the *k*th cycle, the predicted worth *x*_*i*_′(*k*+1) of the *k*+1th cycle task is expressed as

(14) $$\begin{array}{c} x_{i}^{\prime }\left(k+1\right)=a_{i}^{\prime }\left(k\right)+b_{i}^{\prime }\left(k\right)+c_{i}^{\prime }\left(k\right). \end{array}$$

The parameters *a*_*i*_′(*k*), *b*_*i*_′(*k*), and *c*_*i*_′(*k*) are, respectively, as follows:

(15) $$\begin{array}{c} a_{i}^{\prime }\left(k\right)=3p_{i}^{1}\left(k\right)-3p_{i}^{2}\left(k\right)+3p_{i}^{3}\left(k\right),\\ b_{i}^{\prime }\left(k\right)=\frac{a}{2{\left(1-a\right)}^{2}}\left[\left(6-5a\right)p_{i}^{1}-2\left(5-4a\right)p_{i}^{2}\left(k\right)+\left(4-3a\right)p_{i}^{3}\left(k\right)\right],\\ c_{i}^{\prime }\left(k\right)=\frac{a^{2}}{2{\left(1-a\right)}^{2}}\left[p_{i}^{1}\left(k\right)-2p_{i}^{2}\left(k\right)+p_{i}^{3}\left(k\right)\right]. \end{array}$$

In the formula, *p*_*i*_^1^(*k*) is the first smoothing value, *p*_*i*_^2^(*k*) is the second smoothing value, *p*_*i*_^3^(*k*) is the third smoothing value, and the calculation formula is as follows:

(16) $$\begin{array}{c} p_{i}^{1}\left(k\right)=ax_{i}\left(k\right)+\left(1-a\right)p_{i}^{1}\left(k-1\right), \end{array}$$

(17) $$\begin{array}{c} p_{i}^{2}\left(k\right)=ax_{i}\left(k\right)+\left(1-a\right)p_{i}^{2}\left(k-1\right), \end{array}$$

(18) $$\begin{array}{c} p_{i}^{3}\left(k\right)=ax_{i}\left(k\right)+\left(1-a\right)p_{i}^{3}\left(k-1\right). \end{array}$$

Equations (16)–(18) are the first smoothing process, the second smoothing process, and the third smoothing process separately, where *x*_*i*_(*k*) is the practical workload value of the task_*i*_ task type in the *k*th cycle, which is the smoothing coefficient, namely, between (0.1). To perform a cubic exponential smoothing method, pay attention to the choice of primary values *p*_*i*_^1^(0), *p*_*i*_^2^(0), and *p*_*i*_^3^(0). It can usually be replaced by the average of the previous measurements, or it can be replaced directly by the first cycle reading, which in this chapter can be replaced by the first cycle reading. The analysis shows that any smoothed predicted value is obtained by correcting the original predicted value for the prediction error. Size indicates the size of the correction. The larger the value, the wider the correction range, and vice versa.

## 4. Analysis and Prediction of the Influence Factors of Green Computing on the Carbon Cycle Process in Smart Cities

### 4.1. Analysis of Carbon Storage in Smart Cities

From the view of the composition of carbon storage, smart city carbon pools can be divided into two categories: natural carbon pools and anthropogenic carbon pools, of which natural carbon pools account for about 85% of the total carbon stock, and anthropogenic carbon pools account for a relatively small proportion, accounting for only 15%. It can be found out from Figure 3 that the increase in overall carbon storage is relatively slow, from 67.82 million tons in 2007 to 70.05 million tons in 2019, and the natural carbon pool increases from 2007 to 2019. There is no significant difference in the total amount of savings, which has been around 60 million tons; it can be found out from Figure 4 that the amount of anthropogenic carbon storage has been increasing year by year, from 7.82 million tons in 2007 to 9.98 million tons in 2019. The proportion is also rising slowly, from 11.53% in 2007 to 14.25% in 2019, which shows that although the total amount of anthropogenic carbon storage is not large, with the development of urbanization, a large amount of carbon-containing substances contribute, especially the carbon storage capacity of buildings and green cities gradually increases, producing anthropogenic carbon in preparation for further accumulation. The results suggest that, in addition to the naturally important carbon storage, anthropogenic carbon storage is an important way of storing carbon in urban systems, which is partly affected by global warming as shown in Figures 3 and 4.

From Table 1, it can be seen that in the composition of carbon pools, soil accounts for the largest proportion, accounting for about 82% of the total, followed by housing construction, accounting for about 5% of the total, forest land accounting for about 4.6% of the total, and urban greening about 3.80% of the total, commercial buildings about 2.7% of the total, others about 1% of the total, furniture about 0.56% of the total, and books about 0.34% of the total.

### 4.2. Analysis of Influence Factors of Green Computing on Carbon Cycle Process in Smart City

From Table 2 and Figure 5, it can be found out that the overall contribution value of each factor (10^4^ tC) is the largest in 2018–2019, the value of ΔC is 1635.06*∗*10^4^ tC, and the dedication value of the industrial carbon emission intensity factor is −346.7*∗*10^4^ tC, the dedication value of the industrial structure effect factor is 23.63*∗*10^4^ tC, the dedication value of the economic growth element is 1716.24*∗*10^4^ tC, and the contribution value of the population factor is 241.89*∗*10^4^ tC; the smallest is 2009–2010, ∆C is 1.5*∗*10^4^ tC, the contribution value of the industrial carbon emission intensity factor is −84.09*∗*10^4^ tC, the dedication value of the industrial structure effect factor is −19.29*∗*10^4^ tC, and the dedication value of the economic growth element is 90.16*∗*10^4^ tC. The contribution value of the population factor is 14.71*∗*10^4^ tC. The largest contribution factor is the economic development factor, and the smallest factor is the industrial carbon emission intensity factor. The overall contribution rate of each factor is the largest in 2018–2019. The value of *D* is 2.65, the industrial carbon intensity index contribution index is 0.92, the industrial structure effect index contribution index is 0.98, the economic development index contribution index is 1.1, and the population index contribution index is 1.02. The proportion of factors is 0.81, the industrial structure effect factor is 1.01, the economic development factor is 2.78, and the population factor is 1.16. The main positive factors affecting the significant increase in carbon dioxide emissions from smart cities from 2010 to 2019 are economic development factors and demographic factors, of which economic development factors, namely, GDP per capita, have the greatest impact on the increase in carbon dioxide emissions. The total emissions are less than the increase in the overall CO2 emissions, and the remaining years are greater than the total changes in CO2 emissions. This suggests that the total increase in CO2 emissions from smart cities could have been greater if economic development had not had a dampening effect on CO2 emissions from other factors. Demographic factors have a positive (long-term) influence on the increase in annual CO2 emissions, but overall, the contribution is not of much value.

The main positive elements for the substantial increase in carbon emissions in smart cities from 2010 to 2019 are economic development factors and population factors. Among them, the economic development factor, namely, GDP per capita, has the greatest driving influence on the development of carbon emissions. The contribution of total emissions was lower than the increase in overall carbon emissions, and the rest of the years were higher than the overall change in carbon emissions.

Figure 6 shows that the trend line for economic development factors was consistently higher than other factors from 2011 to 2019. From 2011 to 2015, the contribution rate of economic factors to the change of carbon dioxide emissions was lower than that of the overall carbon dioxide emissions, and carbon dioxide increased first and then decreased, so the change rate of economic factors to carbon dioxide emissions development factors exceeded the overall indicators for 2015–2018. The industrial CO2 emission index, industrial structure effect, and population index are always at the low end of the total value. Since the total efficiency is the product of the contribution factors of each factor, the contribution factor of each factor is greater than 1, indicating that it contributes to the increase in CO2 emissions; if the premium is less than 1, it is an inhibitory factor. It can be seen that the economic development factor has the greatest impact on the increase of carbon dioxide emissions, and its share is even greater than the overall change rate of carbon dioxide emissions.

It can be seen in Table 3 that at the 5% significant level, the *P* values between GDP (100 million yuan), population (10,000 people), built-up area (km^2^), and carbon emissions are all less than 0.05, indicating that the path of variables and carbon emissions has a significant impact. *R*^2^ = 0.972, and through the 1% significance test, the results show that it is more in line with the relationship between CO2 emissions and influencing factors. The main determinants of CO2 emissions are the growth of economic scale, the growth of the average daily population, and the increase of built-up space. Overall, economic growth stimulates industrial production and energy consumption, mainly through fossil fuels, as the main driver of growth in CO2 emissions; population growth increases CO2 emissions from food, household energy needs, energy consumption for passenger transport, and construction on the ground. In the process, the expansion of the construction industry has increased the energy demand and CO2 emissions of the building industry, which have become the main drivers of urban CO2 emissions. In addition, the equation can be used to predict total smart CO2 emissions.

In the adaptation index, the fitting value of CMIN/DF is 2, and the critical value is less than 5, so the judgment result is in line; the fitting value of GFI is 0.98, the fitting value of AGFI is 1.01, and the fitting value of RFI is 1.12, all meet the critical value greater than 0.9, so the judgment result is consistent; the PNFI external fitting value is 1.89, and the critical value is greater than 0.5, so the judgment result is consistent; the RMSEA fitting value is 0.42, and the critical value is less than 0.08, so the judgment result is in line. It shows that the model fitting effect is good, and the model is established as shown in Table 4.

### 4.3. Prediction of Carbon Cycle Process by Green Computing in Smart Cities

It can be seen from Figure 7 that the difference between the actual value trend line and the predicted value trend line is not large, indicating that the error between the actual value and the predicted value is small, and the predicted result is reliable. In 2011, the actual value of carbon emissions was 68.8 million tons, and the predicted value was 68.01 million tons; in 2012, the actual value of carbon emissions was 69.02 million tons, and the predicted value was 69.2 million tons; in 2013, the actual value of carbon emissions was 69.2 million tons. In 2014, the actual value of carbon emissions was 69.26 million tons, and the predicted value was 69 million tons; in 2015, the actual value of carbon emissions was 69.46 million tons and the predicted value was 69.50 million tons. In 2016, the actual value of carbon emissions was 69.69 million tons, and the predicted value was 70 million tons; in 2017, the actual value of carbon emissions was 69.8 million tons, and the predicted value was 69.78 million tons; in 2018, the actual value of carbon emissions is 69.88 million tons, and the predicted value is 69.91 million tons; in 2019, the actual value of carbon emissions is 70.05 million tons, and the predicted value is 70.21 million tons.

From Table 5, it can be found out that the forecasted carbon emission value from 2020 to 2028 is slowly adding year by year. The predicted value of CO2 emissions in 2022 is 13.82 million tons, the predicted value of CO2 emissions in 2023 is 14.27 million tons, the predicted value of CO2 emissions in 2024 is 14.68 million tons, the predicted value of CO2 emissions in 2025 is 14.68 million tons, and The predicted value of CO2 emissions in 2026 is 15.62 million tons, the predicted value of CO2 emissions in 2027 is 15.73 million tons, and the forecasted value of CO2 emissions in 2028 is 15.92 million tons.

## 5. Conclusion

For the progress of human society, “low carbon” must be “relatively low carbon” to ensure development rather than “reducing carbon emissions” regardless of cost or expense. Therefore, future development should take into account the “total” land use and evaluate the comprehensive benefits of land use and their regulation: on the one hand, ecological benefits and the effect of reducing CO2 emissions from land use, and on the other hand, it should consider improving people's lives, society, and economic benefits, which require further evaluation and consideration to find the best combination. Create an ecologic civilization publicity and education system, strengthen publicity and education, enhance social consciousness of ecological environmental conservation, and increase the enthusiasm of society to participate in ecological environmental protection. Advocate green and low-carbon life, accelerate the transformation of lifestyle and consumption patterns to uncomplicated, alleviative, green and low-carbon, civilized and healthy; they advocate green travel, green consumption, low-carbon, and moderate consumption and oppose debauchery and waste. Please pay attention to garbage disposal when eating, advocate garbage sorting and recycling, and do not pollute the environment. Carry out the creation of green brands, for example, green schools, green institutions, green hotels, green hospitals, and green communities; use brands to attract public opinion; improve environmental awareness and the concept of ecological civilization; and consciously shape social trends to care for and protect the environment.

## Figures and Tables

**Figure 1:** The main components of the smart city ecosystem.

**Figure 2:** The relationship between the functions, patterns, and roles of smart city systems and carbon emissions.

**Figure 3:** Changes in trend of total carbon storage in smart city eco-economic system.

**Figure 4:** Changes in anthropogenic carbon pools and their proportions in smart cities over the years.

**Figure 5:** Contributions of various factors to changes in carbon emissions in smart cities over the years.

**Figure 6:** Contribution rate of various factors in the change of carbon emissions in smart cities over the years.

**Figure 7:** Comparison of actual and predicted smart city values.

**Table 1:** Composition analysis of smart city carbon pool.

Constitute	Soil (%)	Construction (%)	Woodland (%)	City greening (%)	Commercial building (%)	Books (%)	Furniture (%)	Other (%)
Proportion	82	5	4.60	3.80	2.70	0.34	0.56	1.00

**Table 2:** Elements decomposition analysis of changes in overall carbon emissions in smart cities.

Year	Contribution of each factor (10^4^ tC)					Each factor index					
	Industrial carbon emission intensity factors	Industrial structure effect	Economic development factors	Population factor	Overall	Industrial carbon emission intensity factors	Industrial structure effect	Economic development factors	Population factor	Overall
	Δ*C*_*f*_	Δ*C*_*sf*_	Δ*C*_*g*_	Δ*C*_*p*_	Δ*C*	*D*_*f*_	*D*_*s*_	*D*_*g*_	*D*_*p*_	*D*
2009–2010	−84.09	−19.29	90.16	14.71	1.5	0.92	0.98	1.1	1.02	1
2010–2011	−48.48	−11.77	104.18	18.76	52.69	0.95	0.99	1.11	1.02	1.06
2011–2012	31.95	15.08	143.36	18.21	208.35	1.03	1.01	1.13	1.02	1.2
2012–2013	1.01	42.67	194.5	27.27	265.47	1	1.03	1.15	1.02	1.21
2013–2014	145.03	21.94	208.73	35.7	411.22	1.08	1.01	1.13	1.03	1.27
2014–2015	−141.55	7.48	242.87	38.23	147.03	0.93	1	1.13	1.02	1.08
2015–2016	−124.11	28.51	277.38	35.62	217.38	0.94	1.01	1.14	1.02	1.1
2016–2017	−153.71	−35.15	236.09	27.38	74.71	0.93	0.99	1.11	1.01	1.03
2017–2018	9.31	−37.33	253.58	21.16	246.71	1	0.96	1.11	1.01	1.1
2018–2019	−346.7	23.63	1716.24	241.89	1635.06	0.81	1.01	2.78	1.16	2.65

**Table 3:** Regression parameter analysis of influencing factors of carbon emissions.

	Standardized estimates	Standard deviation	Critical ratio	*P* value
GDP (100 million yuan)	−0.144	0.2	12.34	0.02
Population (10,000 people)	32.12	0.3	23.14	0.06
Built-up area (km^2^)	−1.05	0.12	26.45	0.05

**Table 4:** Overall model fitting results.

Adaptation indicator	CMIN/DF	GFI	AGFI	RFI	PNFI	RMSEA
Critical value	<5	>0.9	>0.9	>0.9	>0.5	<0.08
Fitted value	2	0.98	1.01	1.12	1.89	0.42
Judgment result	Meets	Meets	Meets	Meets	Meets	Meets

**Table 5:** 2020–2028 CO2 emission forecast.

Year	Predicted value (10,000 tons)
2020	1220
2021	1327
2022	1382
2023	1427
2024	1468
2025	1503
2026	1562
2027	1573
2028	1592

## Data Availability

The experimental data used to support the findings of this study are available from the corresponding author upon request.
